The article "Polysaccharide IV from Lycium barbarum L. Improves Lipid Profiles of Gestational Diabetes Mellitus of Pregnancy by Upregulating ABCA1 and Downregulating Sterol Regulatory Element-Binding Transcription 1 via miR-33" was retracted in 2023. Reasons: concerns about the data; concerns about the images.

# Polysaccharide IV from *Lycium barbarum L*. Improves Lipid Profiles of Gestational Diabetes Mellitus of Pregnancy by Upregulating ABCA1 and Downregulating Sterol Regulatory Element-Binding Transcription 1 *via* miR-33

**DOI:** 10.3389/fendo.2018.00049

**Published:** 2018-02-23

**Authors:** Shuli Yang, Lihui Si, Limei Fan, Wenwen Jian, Huilin Pei, Ruixin Lin

**Affiliations:** ^1^Department of Gynecology and Obstetrics, The Second Hospital of Jilin University, Changchun, China; ^2^Department of Hepatobiliary and Pancreatic Surgery, The Second Hospital of Jilin University, Changchun, China

**Keywords:** *Lycium barbarum L.*, gestational diabetes mellitus, ATP-binding cassette transporter A1, sterol regulatory element-binding transcription, miR-33

## Abstract

*Lycium barbarum L*. (LBL) has beneficial effects on gestational diabetes mellitus (GDM) but the related mechanism remains unclear. Polysaccharides of LBL (LBLP) are the main bioactive components of LBL. miR-33, ATP-binding cassette transporter A1 (ABCA1) and sterol regulatory element-binding transcription 1 (SREBF1) affect lipid profiles, which are associated with GDM risk. LBLP may exert protective against GDM by affecting these molecules. Four LBLP fractions: LBLP-I, LBLP-II, LBLP-III, and LBLP-IV were isolated from LBL and further purified by using DEAE-Sephadex column. The effects of purified each fraction on pancreatic beta cells were comparatively evaluated. A total of 158 GDM patients were recruited and randomly divided into LBL group (LG) and placebo group (CG). miR-33 levels, lipid profiles, insulin resistance and secretory functions were measured. The association between serum miR-33 levels and lipid profiles were evaluated by using Spearman’s rank-order correlation test. After 4-week therapy, LBL reduced miR-33 level, insulin resistance and increased insulin secretion of GDM patients. LBL increased the levels of ABCA1, high-density lipoprotein cholesterol (HDL-C) and reduced miR-33, SREBF1, low-density lipoprotein cholesterol (LDL-C), total cholesterol (TC), triglyceride (TG), and malondialdehyde. Homeostatic model assessment of β-cell function and insulin resistance was lower in LG than in CG, whereas homeostatic model assessment of β-cell function and insulin secretory function was higher in LG than in CG. There was a strong positive association between miR-33 level and TG, or TC and or LDL-C, and a strong negative association between miR-33 level and HDL-C. The levels of miR-33 had negative relation with ABCA1 and positive relation with SREBF1. ABCA1 has negative relation with TG, TC, and LDL-C and positive relation with HDL-C. Inversely, SREBF1 had positive relation with TG, TC, and LDL-C and negative relation with HDL-C. The main bioactive compound LBLP-IV of LBL increased insulin secretion of beta cells and the levels of ABCA1, and reduced miR-33 levels and SREBF1 in beta cells. However, LBLP-IV could not change the levels of these molecules anymore when miR-33 was overexpressed or silenced. LBLP-IV had the similar effects with LBL on beta cells while other components had no such effects. Thus, LBLP-IV from LBL improves lipid profiles by upregulating ABCA1 and downregulating SREBF1 *via* miR-33.

The article "Polysaccharide IV from Lycium barbarum L. Improves Lipid Profiles of Gestational Diabetes Mellitus of Pregnancy by Upregulating ABCA1 and Downregulating Sterol Regulatory Element-Binding Transcription 1 via miR-33" was retracted in 2023. Reasons: concerns about the data; concerns about the images.

## Introduction

Gestational diabetes mellitus (GDM), a special type of diabetes, is caused by multiple factors with genetic predisposition (1) and endocrine metabolic diseases (2, 3). GDM is defined as the different glucose intolerance that occurs within the first trimester of pregnancy. It is estimated that the incidence of GDM represents average 3–8% of all pregnancies (4). GDM incidence will continue to increase due to the changes of lifestyle and living conditions. Compared with other types of diabetes mellitus, GDM not only affects their own health status and but also increases the risk of postpartum diabetes. Previous study showed that the cumulative incidence of type 2 diabetes mellitus was 6 weeks to 28 years in postpartum women with GDM (5). GDM has negative effects on future generations, including neonatal death (6), stillbirth (7), perinatal mortality (8), preeclampsia (9), large fetus (10), neonatal jaundice (11), low blood sugar (12), low calcium (13), and so on. However, the pathogenesis of GDM is still not fully understood. Many countries have invested much money on the research programs of GDM, including GDM pathogenesis, impact factors and diagnostic criteria. Living environment (14), family history (15), pregnancy (16, 17), low birth weight (18), prepregnancy obesity (19), and dietary imbalance (20, 21) are common risk factors of GDM. Balanced nutrition and appropriate physical labor and exercise are the main methods for preventing the occurrence of GDM (22).

Medical treatment is still the main method for GDM therapy (23, 24). However, the safety or efficacy of the medicine remains unclear in pregnancy (25, 26). It is necessary to find natural medicine with a fewer side effects. *Lycium barbarum L*. (LBL) is a deciduous woody perennial plant primarily in the Ningxia Hui Autonomous Region (Ningxia, China) (27). Polysaccharides of LBL (LBLP) are the main bioactive components (28, 29). LBLP-IV administration has been reported to control the animal model with diabetes. LBLP-IV may be a potential therapeutic agent in diabetic treatment (30). However, the molecular mechanism for the effects of LBLP-IV on diabetes remains unknown. MicroRNA is short, single-stranded RNA molecules with 22 nucleotides in length. MiR-33 can regulate lipid metabolism (31), which is associated with GDM. There is much evidence linking miR-33 to lipid metabolism by targeting ATP-binding cassette transporter A1 (ABCA1) and sterol regulatory element-binding transcription 1 (SREBF1) (32). ABCA1 is the cholesterol efflux regulatory protein, which regulates cholesterol efflux and phospholipid homeostasis (33). SREBP are the transcription factors, which bind to the sterol regulatory element and repressed its expression, including ABCA1 gene (34). ABCA1 (35) and SREBF1 (36) affect lipid metabolism too. Thus, the polysaccharides may improve lipid profiles by affecting ABCA1 and SREBF1 levels *via* miR-33. However, the miR-33-related molecular mechanisms for the functions of LBL on GDM patients are still unclear.

The article "Polysaccharide IV from Lycium barbarum L. Improves Lipid Profiles of Gestational Diabetes Mellitus of Pregnancy by Upregulating ABCA1 and Downregulating Sterol Regulatory Element-Binding Transcription 1 via miR-33" was retracted in 2023. Reasons: concerns about the data; concerns about the images.

In this study, we want to explore the effects of LBL on GDM patients by investigating serum lipid profiles and related molecules. Changes in the miR-33, ABCA-1, and SREBF1 expressions, as well as insulin sensitivity and blood insulin and resistin levels, were also assessed. Meanwhile, the bioactive compound from LBL was isolated and its effects on β cell were measured.

## Materials and Methods

### LBL Polysaccharides Isolation

*Lycium barbarum L*. leaves were purchased from Ningxia, China and LBL polysaccharides were isolated according to an early report (37). Fifty-microgram LBL leaves were crushed to fine powder and extracted in triplicate by using 1 l distilled water for 1 h at 90°C. The filtrated solution was concentrated by using a rotary evaporator (RE-52A, Shanghai Woshi Co., Shanghai, China) at 55°C, and precipitated by adding fourfold volume of anhydrous ethanol. LBLP were washed three times with anhydrous ethanol and acetone after being centrifuged at 3,000 rpm for 15 min, and then and finally lyophilized. The crude protein was removed by using the Sevag method (38) and decolorized with the macroreticular resin AB-8 (Cangzhou Resin Company, Cangzhou, Hebei, China). Final polysaccharides were isolated by using a DEAE SephadexA-25 column (Amersham Pharmacia Biotech, Piscataway, NJ, USA) equilibrated with distilled water for one day. Individual polysaccharide was eluted with distilled water, 0.1 and 0.2 M NaCl at 0.8 mL/min. The polysaccharide fractions were collected at 2 min/tube using an automatic collector (Beijing Xinhuizeao Technology Co., Ltd., Beijing, China), then the collected solution was dialyzed (MWCO 3600, Sigma) and lyophilized finally.

The homogeneity of isolated polysaccharide was determined by high-performance gel-permeation chromatography (HP-GPC) (Dionex, Sunnyvale, CA, USA). Twenty-microliter sample solution was performed at a flow rate of 0.5 mL/min (distilled water and 100, 200 mM NaCl) as a mobile phase. The columns were calibrated with T-series dextran (T-10, 40, 70, 500, 2,000), and the molecular weight of polysaccharides was confirmed by referencing to a calibrated curve.

The article "Polysaccharide IV from Lycium barbarum L. Improves Lipid Profiles of Gestational Diabetes Mellitus of Pregnancy by Upregulating ABCA1 and Downregulating Sterol Regulatory Element-Binding Transcription 1 via miR-33" was retracted in 2023. Reasons: concerns about the data; concerns about the images.

### Participants

All protocols were approved by ethical committee of our hospital (Approval no. 201602X4), and the study was carried out according to the principles described in the World Medical Association Declaration of Helsinki (39). All subjects gave written informed consent in accordance with the Declaration of Helsinki. From April 2016 to May 2016, a total of 158 women diagnosed with GDM were collected at our hospital. All the pregnant women met the diagnostic criteria of GDM *via* a 2-h 75-g oral glucose tolerance test according to an earlier report (40).

### Including Criteria

Pregnant women were age 18–40 years; the patient had singleton pregnancy and no previous GDM; pregnant women had an impairment of their glucose tolerance according to the results of a 2-h 75-g oral glucose tolerance test; the patients were diagnosed with GDM from 26 to 30 weeks of gestation.

### Excluding Criteria

The patients were smokers and or alcohol drinkers; some condition and or medication that affected glucose levels; the patients were unwilling to follow the prescribed diet. The patients had cardiac, dizziness, and related diseases; the patients had obvious abnormal clinical findings.

### GDM Patients Grouping

After screening *via* inclusion and exclusion criteria, 158 patients were evenly and randomly assigned into a LBL group (LG, received 10-mg LBL daily) and a control group (CG, received 10-mg placebo daily) (Figure 1).

**Figure 1:** Flowchart of the study population. ABCA1, ATP-binding cassette transporter A1. SREBF1, sterol regulatory element-binding transcription. The whole period was 4 weeks.

### Blood Glucose (BG) Measurement

Five-milliliter blood is either directly sucked into a vacuum test tube from a vein of each patients. Serum was isolated by centrifugation at 10,000 rpm for 5 min. The concentration of BG was measured by using glucose oxidase (41). Unified quality control standards were used for all the 26–30-week pregnancy with GDM. Fasting blood glucose (FBG) was measured in the morning *via* centrifugation after taking venous blood from each subject, and then dissolved in two pairs of bottles filled with water.

### Biochemical Analysis

The concentrations of glucose and HbAlc were measured after taking 2-h 75 g oral glucose. The concentration of BG was measured by using glucose oxidase (41). Serum HbA1c levels were measured by was measured by HPLC (D-10 Dual Program; Bio-Rad, Hercules, CA, USA). High- and low-density lipoprotein-cholesterol (HDL-C and LDL-C) were measured by using an Olympus AU 600 auto-analyzer (Olympus Optical Co. Ltd., Schimatsu-Mishima, Japan). Triglyceride (TG) levels were measured a Technicon RA-500 analyzer (Bayer, Etobicoke, ON, Canada). Basal BG and FBG levels were examined by ABL 800FLEX blood gas analyzer (Midland, ON, Canada). Serum resistin was measured by using the resistin ELISA kit from Phoenix Pharmaceuticals (Belmont, CA, USA) according to manufacturer’s instructions. Serum basal insulin and fasting insulin (FINS) were tested by radioimmunoassay (Linco, Seaford, DE, USA). Homeostatic model assessment of β-cell function and insulin resistance (HOMA-IR) and homeostatic model assessment of β-cell function and insulin secretory function (HOMA-IS) were measured by using the following equations: HOMA-IR = FBG × FINS/22.5 and HOMA-IS = 20 × FINS/(FBG − 3.5), respectively.

The article "Polysaccharide IV from Lycium barbarum L. Improves Lipid Profiles of Gestational Diabetes Mellitus of Pregnancy by Upregulating ABCA1 and Downregulating Sterol Regulatory Element-Binding Transcription 1 via miR-33" was retracted in 2023. Reasons: concerns about the data; concerns about the images.

### Measurement of Serum Lipid Profiles

Two-milliliter serum was separated from whole blood by allowing the blood to just let stand. A lipid profiles is closely associated with the risk of GDM (42–44). Lipid profiles were measured by using the same method in Section “MiR-33 Silencing.” Malondialdehyde (MDA) level was measured by using a MDA detection kit (A003; Nanjing Jiancheng Bioengineering Institute, Nanjing, China). Lipid indexes were measured before and after 4-week experiment.

### Cell Culture

Gestational diabetes mellitus represents the major diabetes, and β-cell dysfunction plays an important role in the development and progression of the disease. The components purified by DEAE-Sephadex A-25 column, were measured by using human pancreatic carcinoma cell SW1990, which was purchased from cell bank, CAS (Shanghai, China). The cell lines were cultured in RPMI-1640 at 37°C with 5% CO_2_. After 3-day culture, the cell concentrations were adjusted to 1 × 10^5^ cells/mL and 100 µL cells were transferred to each cell of 96-cell plate, treated with 10 µg/mL different fractions and further cultured for three days under the same situation.

### MiR-33 Silencing

Lipofectamine™ 2000 (Invitrogen, Waltham, MA, USA) was used to transfect islet β-cell line SW1990 with miR-33 RISC complex. 10^5^ SW1990 cells were seeded in six-well plates. Scrambled control siRNA was carried out (Beijing Dingguo Changsheng Biotechnology, Beijing, China). miR-33 (GenBank No., NR_029507.1) four target siRNA sequences: UGUGGUGCAUUGUAGUUGCAUUGCA, UGGUGCAUUGUAGUUGCAUUGCAUG, GCAUUGUAGUUGCAUUGCAUGUUCU and CAUUGUAGUUGCAUUGCAUGUUCUG. The transfection with 40 nM siRNA was performed in DMEM (with 1% l-glutamine, 10% FCS and without penicillin/streptomycin) for 72 h.

The article "Polysaccharide IV from Lycium barbarum L. Improves Lipid Profiles of Gestational Diabetes Mellitus of Pregnancy by Upregulating ABCA1 and Downregulating Sterol Regulatory Element-Binding Transcription 1 via miR-33" was retracted in 2023. Reasons: concerns about the data; concerns about the images.

### The Effects of LBL Fractions on Insulin Secretion in SW1990 Cells

SW1990 were seeded in 24-well plates (1 × 10^5^ cells/well), treated with different fractions of LBL and cultured for 3 days to investigate insulin secretion. Insulin level was measured by using an insulin ELISA kit (Thermo Fisher Scientific Inc., Cleveland, OH, USA). After the determination of bioactive components, LBL was then used for clinical trials.

### Quantitative RT-PCR Analysis

Blood samples were obtained from GDM patients. Serum was isolated from blood samples within 2 h. Total RNA was extracted by using a miRNeasy Serum/Plasma Kit (QIAGEN Sciences, Germantown, MD, USA). Finally, 2-µg RNA was obtained from 1-mL serum. MiR-33 (GenBank No. NR_029507.1), forward primer: 5′-GTCCGTGGTGCATTGTAGT-3′; reverse primer: 5′-GTGCAGGGTCCGAGGT-3′. U6 (GenBank No. NR_004394.1), forward primer: 5′-TTGGTGCTCGCTTCGGCA-3′; reverse primer: 5′-GTGCAGGGTCCGAGGT-3′. U6 snRNA was used as an internal control. ABCA1 (GenBank No. AB055982.1), forward primer: 5′-ATTGTGGCTCGCCTGTTCTC-3′; reverse primer: 5′-TAGACTTTGGGAGAGAGAGG-3′. SREBF1 (GenBank No. NM_001005291.2), forward primer: 5′-TGAGCTCCTCTCTTGAAGCC-3′; reverse primer: 5′-GTAGCCTAACACAGGGGTGG-3′; Beta actin (GeanBank No. HQ154074.1, as a loading control), forward primer: 5′-TCCAGCCTTCCTTCCTGGGC-3′; reverse primer: 5′-GCCAGGGTACATGGTGGTAC-3′. qRT-PCR was conducted by using an Applied Biosystems 7300 Real-time PCR System. 1-µL RT products were added to 20-µL reaction volume including 0.5-µL sense primer and reverse primer, 1-µL SYBR^®^ Green Real-Time PCR Master Mixes (Thermo Fisher Scientific, Waltham, MA, USA), and one-unit Taq [Takara Biotechnology (Dalian) Co., Ltd., Dalian, China]. The reaction was carried out by using the following parameters: 94°C for 5 min, followed by 45 cycles of 94°C for 20 s and 65°C for 1 min. After the reaction, the CT was calculated *via* threshold settings. The ratio of uterine sarcoma serum miRNA and healthy subjects was presented by using 2 ^− ΔG^, in which ΔG = C_T cancer_ − C_T normal_.

### Western Blot Analysis

SW1990 cell lines were treated with cocktail and lysed *via* a freezing and thawing method. Meanwhile, serum samples were also prepared for Western Blot analysis. Twenty-five microgram proteins were separated by 12% SDS-PAGE and transferred to a PVDF membrane, which was blocked by non-fat milk for 30 min. The membranes were incubated with the antibodies ABCA1 (ab66217) and SREBF1 (ab28481), Beta actin (ab6276, as a loading control), goat polyclonal secondary antibody to rabbit IgG-H&L (HRP) (ab6721, Abcam, Cambridge, MA, USA). With X-ray film exposure, the expression of ABCA1 and SREBF1 was detected *via* Quantity One software.

The article "Polysaccharide IV from Lycium barbarum L. Improves Lipid Profiles of Gestational Diabetes Mellitus of Pregnancy by Upregulating ABCA1 and Downregulating Sterol Regulatory Element-Binding Transcription 1 via miR-33" was retracted in 2023. Reasons: concerns about the data; concerns about the images.

### Statistical Analysis

Results were presented as the mean ± SEM. Paired student’s *t*-test was used to compare the differences between two groups. Spearman’s rank-order correlation test was used to test the relationship between two variables. There were statistically significant differences if *P* < 0.05.

## Results

### Characterization of LBL

Four main polysaccharides were isolated from LBL after the purification of DEAE-Sephadex A-25 column (Figure 2A), which was accordant with an earlier report (37). The isolated components were further confirmed by HP-GPC under the conditions that produced masses predicted for LBLP I (Figure 2B), LBLP II (Figure 2C), LBLP III (Figure 2D), and LBLP IV (Figure 2E) were 55.2, 94.0, 241.3, and 418.0 kDa, respectively.

**Figure 2:** The polysaccharides of the extracts of *Lycium barbarum L*. (LBL) are purified by using a DEAE SephadexA-25 column. **(A)** There are four main polysaccharides [polysaccharides of LBL (LBLP) I, II, III, and IV] in the extracts of LBL **(B)** High-performance gel-permeation chromatography (HP-GPC) analysis of LBLP I. **(C)** HP-GPC analysis of LBLP II. **(D)** HP-GPC analysis of LBLP III. **(E)** HP-GPC analysis of LBLP IV.

### Baseline Characters

Table 1 shows the clinical characters were similar between two groups. The mean ages of were at age of 30.1 ± 5.4 in LG and 29.5 ± 4.3 in CG. The statistical difference was insignificant for baseline demographic and metabolic characteristics of the patients between two groups (*P* > 0.05).

**Table 1:** Baseline demographic and metabolic characteristics of GDM (gestational diabetes mellitus of pregnancy) subjects.

Characteristics of patients	LG (*n* = 79)	CG (*n* = 79)	*t*/χ^2^	*P*-value
Age (years)	30.1 ± 5.4	29.5 ± 4.3	0.23	0.64^a^
Race, *n* (%)				
Han Zhu	64	65	0.04	0.84^b^
Manchu	10	9	0.06	0.81^b^
Mongolians	4	4	0.13	0.72^b^
Tibetans	1	1	0.51	0.48^b^
Body weight (kg)	68.3 ± 10.2	67.9 ± 11.5	0.97	0.12^a^
BMI (kg/m^2^)	28.4 ± 4.9	27.7 ± 5.3	0.86	0.25^a^
Insulin (mIU/L)	20.6 ± 2.3	20.5 ± 2.6	0.23	0.69^a^
HbA1c (%)	6.9 ± 1.7	6.7 ± 1.9	0.72	0.58^a^
FBG (mmol/L)	8.3 ± 1.1	8.4 ± 1.2	0.84	0.32^a^
2hPG (mmol/L)	14.9 ± 2.5	14.1 ± 3.2	0.60	0.55^a^
TG (mmol/L)	2.8 ± 1.2	2.7 ± 1.4	0.19	0.81^a^
TC (mmol/L)	5.9 ± 1.4	5.7 ± 1.6	0.24	0.40^a^
HDL-C (mmol/L)	1.3 ± 0.3	1.4 ± 0.5	0.20	0.56^a^
LDL-C (mmol/l)	3.7 ± 1.0	3.9 ± 1.2	0.18	0.72^a^
Resistin (ng/mL)	15.1 ± 4.6	15.2 ± 3.7	1.24	0.15^a^
HOMA-IR	6.4 ± 3.4	6.6 ± 3.5	1.90	0.26^a^
HOMA-IS	66.1 ± 36.7	68. 3 ± 27.4	1.55	0.10^a^

*One hundred and fifty-eight patients were assigned into an LBL group (LG, received 10 mg LBL daily) and a control group (CG, received 10-mg placebo daily). There is not significant statistic difference at *P* > 0.05*.

*^a^Paired t-test*.

*^b^Chi-square test*.

The article "Polysaccharide IV from Lycium barbarum L. Improves Lipid Profiles of Gestational Diabetes Mellitus of Pregnancy by Upregulating ABCA1 and Downregulating Sterol Regulatory Element-Binding Transcription 1 via miR-33" was retracted in 2023. Reasons: concerns about the data; concerns about the images.

*BMI, body mass index. HbA1c, hemoglobin A1c. FBG, fasting blood glucose. 2hPG, 2 h postprandial plasma glucose. TC, total cholesterol. TG, triglyceride; HDL-C, high-density lipoprotein cholesterol. LDL-C, low-density lipoprotein cholesterol; HOMA-IR, homeostatic model assessment of β-cell function and insulin resistance; HOMA-IS, homeostatic model assessment of β-cell function and insulin sensitivity*.

### LBL Consumption Improves Biochemical Parameters and Lipid Pattern

Table 2 shows LBL-reduced insulin resistance and increased insulin sensitivity and secretory function when compared with the CG group (*P* < 0.05). LBL increased the level of HDL-C and reduced the levels of TG, total cholesterol (TC), and LDL-C (*P* < 0.05). The statistical differences were significant for lipid profiles between two groups (*P* < 0.05). Table 3 shows that LBL consumption reduced the serum levels of TG, TC, LDL-C, and MDA while increased the level of HDL-C after 4 weeks. The statistical difference for the changes in the body weight of the patients was insignificant between two groups (LG, 64.9 ± 8.4; CG, 68.7 ± 11.3, *P* > 0.05) after 4-week therapy. The values of HOMA-IR were lower in LG than in CG after therapy when compared with before therapy, whereas the values of HOMA-IS was higher in LG than in CG (*P* < 0.05). All the results suggest that LBL consumption significantly improves lipid patterns of GDM patients, reduces the HOMA-IR and increases the HOMA-IS.

**Table 2:** Parameters changes for antidiabetic activity in both groups.

Parameters	LG (*n* = 79)			CG (*n* = 79)			*P*-values (LG *via* CG)
	Before	After 4 weeks	*P*–values	Before	After 4 weeks	*P*-values	
FBG (mmol/L)	8.3 ± 1.1	8.0 ± 1.3	0.21	8.4 ± 1.2	8.3 ± 1.2	0.17	0.32
2hPG (mmol/L)	14.9 ± 2.5	14.0 ± 3.2	0.16	14.1 ± 3.2	13.9 ± 3.4	0.27	0.30
HbAlc (%)	6.9 ± 1.7	6.4 ± 1.9	0.08	6.7 ± 1.9	6.5 ± 1.6	0.41	0.29
Insulin (mIU/L)	20.3 ± 2.5	52.7 ± 6.8	0.05	20.7 ± 2.4	20.4 ± 2.5	0.34	0.57
Resistin (ng/mL)	15.1 ± 4.6	12.1 ± 3.2	0.02	15.2 ± 3.0	14.5 ± 4.1	0.14	0.03
HOMA-IR	6.4 ± 3.4	5.8 ± 3.1	0.04	6.6 ± 3.5	6.4 ± 2.9	0.17	0.04
HOMA-IS	66.1 ± 36.7	74. 4 ± 21.3	0.03	68. 3 ± 27.4	70.34 ± 14.2	0.24	0.04

*One hundred and fifty-eight patients were assigned into an LBL group (LG, received 10-mg LBL daily) and a control group (CG, received 10-mg placebo daily)*.

**Table 3:** Comparison of lipid pattern in GDM patients before and after therapy.

		Total lipids (g/L)	TG (mmol/L)	TC (mmol/L)	HDL-C (mmol/L)	LDL-C (mmol/L)	MDA (mmol/L)
Before	LG	11.6 ± 1.3	2.8 ± 1.2	5.9 ± 1.4	1.3 ± 0.3	3.7 ± 1.0	1.7 ± 0.3
	CG	11.2 ± 1.1	2.7 ± 1.4	5.7 ± 1.6	1.4 ± 0.5	3.9 ± 1.2	1.6 ± 0.2
	*P*-value	0.45	0.81	0.40	0.56	0.72	0.84
4 weeks	LG	8.2 ± 0.7	1.8 ± 1.2	4.6 ± 1.1	1.6 ± 0.4	3.0 ± 1.2	0.9 ± 0.2
	CG	10.9 ± 1.0	2.6 ± 1.4	5.5 ± 1.0	1.2 ± 0.3	3.9 ± 1.3	1.6 ± 0.4
	*P*-value	0.02*	0.01*	0.02*	0.01*	0.01*	0.01*

*One hundred and fifty-eight patients were assigned into an LBL group (LG, received 10-mg LBL daily) and a control group (CG, received 10-mg placebo daily)*.

The article "Polysaccharide IV from Lycium barbarum L. Improves Lipid Profiles of Gestational Diabetes Mellitus of Pregnancy by Upregulating ABCA1 and Downregulating Sterol Regulatory Element-Binding Transcription 1 via miR-33" was retracted in 2023. Reasons: concerns about the data; concerns about the images.

*P < 0.05 via CG.

*MDA, malondialdehyde*.

### LBL Consumption Reduces Serum miR-33 Level and Relative mRNA Level of SREBPF1, and Increases the Level of ABCA1

The statistical difference was insignificant for relative mRNA levels of miR-33 (Figure 3A), ABCA1 (Figure 3B), and SREBF1 (Figure 3B) between two groups (*P* > 0.05). The serum levels of miR-33 and SREBF1 were decreased while ABCA1 level was increased in LBLG when compared with CG after 4-week LBL consumption (Figures 3A,B, *P* < 0.05). The results suggest that long-term LBL consumption can affect GDM by reducing the serum mRNA levels miR-33 and SREBF1, and increasing the mRNA level of ABCA1.

**Figure 3:** *Lycium barbarum L*. (LBL) consumption significantly reduces miR-33 level and the level of sterol regulatory element-binding transcription 1 (SREBPF1) and increases the level of ABCA1 in gestational diabetes mellitus (GDM) patients. **(A)** The effects of LBL on miR-33 level. **(B)** The effects of LBL on relative mRNA levels of ABCA1 and SREBF1. LG-B, the GDM patients before receiving LBL treatment. CG-B, the GDM patients before receiving placebo. LG-A, the GDM patients after receiving 4-week LBL treatment. CG-A, the GDM patients after receiving 4-week placebo. **(C)** LBL consumption significantly reduces protein level of SREBPF1 and increases the level of ABCA1 in GDM patients. All data were presented as mean values ± SD. There were statistically significant differences if *P < 0.05 vs. a control group.

### LBL Consumption Significantly Reduces Relative Protein Levels of SREBPF1 and Increases the Level of ABCA1

The statistical difference was insignificant for relative protein levels of ABCA1 and SREBF1 among four groups (Figure 3C, *P* > 0.05). The protein level of SREBF1 was decreased and the level of ABCA1 was increased in LG when compared with CG after 4-week LBL consumption (Figure 3C, *P* < 0.05). The results suggest that long-term LBL consumption can affect GDM by reducing protein level of SREBF1, and increasing the protein level of ABCA1.

### MiR-33 Level Is Associated with Lipid Components

Spearman’s Rank-Order Correlation Test showed that the increase in relative level of miR-33 resulted in the increase in the concentrations of TG (Figure 4A), TC (Figure 4B), and LDL-C (Figure 4D) and decrease in the concentration of HDL-C (Figure 4C). There was a strong positive association between miR-33 level and TG, or TC and or LDL-C, and a strong negative association between miR-33 level and HDL-C (*P* < 0.05). These results suggest there is a strong association between serum miR-33 level and lipid components.

The article "Polysaccharide IV from Lycium barbarum L. Improves Lipid Profiles of Gestational Diabetes Mellitus of Pregnancy by Upregulating ABCA1 and Downregulating Sterol Regulatory Element-Binding Transcription 1 via miR-33" was retracted in 2023. Reasons: concerns about the data; concerns about the images.

**Figure 4:** The analysis of spearman’s rank correlation coefficient for the relationship between serum miR-33 level and serum lipid profiles. **(A)** The relationship between serum miR-33 level and triglyceride (TG) concentrations. **(B)** The relationship between serum miR-33 level and total cholesterol (TC) concentrations. **(C)** The relationship between serum miR-33 level and high-density lipoprotein cholesterol (HDL-C) concentrations. **(D)** The relationship between serum miR-33 level and low-density lipoprotein cholesterol (LDL-C) concentrations. Spearman’s Rho is used to measure the strength of association between two variables, where the value *r* falls between 0.5 and 1 means a strong positive correlation and the value *r* falls between −1 and −0.5 means a strong negative correlation.

### Effects of LBLP IV on Insulin Secretion

As shown in Figure 5, LBP IV increased insulin secretion from 20.6 ± 2.6 ng/mL (basal levels) to 52.7 ± 6.8 ng/mL. Under the same situations, LBLP I, II, and III could not cause significant changes for insulin secretion in SW1990 cells. The results suggest that LBLP IV may be the major bioactive ingredient of LBL for the therapy of GDM patients.

**Figure 5:** Polysaccharides of *Lycium barbarum L*. (LBL) activate insulin secretion in SW1990 cells. Values were represented as the means ± SD. from eight experiments. There were statistically significant differences if *P < 0.05. LBL, the extracts of *LB*L with four main polysaccharides (LBLP I, II, III, and IV).

### LBLP IV from LBL Significantly Reduces miR-33 Level, and Relative mRNA Level of SREBPF1, and Increases the Level of ABCA1

To explore the specific function of LBL components, four polysaccharides were purified and tested to their effects on human pancreatic carcinoma cell SW1990. Real time qRT-PCR showed that LBLP I could not affect miR-33 levels (Figure 6A, *P* > 0.05) while LBLP II and III increased miR-33 level, and LBLP IV and LBL reduced miR-33 level significantly (*P* < 0.05) when compared with controls. On the other hand, LBLP I, II and III reduced while LBL and LBLP IV increased relative mRNA levels of ABCA1 (Figure 6B, *P* < 0.05). Comparatively, LBL and LBLP IV reduced more relative mRNA levels of SREBF1 than other polysaccharides (Figure 6B, *P* < 0.05). There were no changes for miR-33 levels when the cells were transfected with scrambled miRNA when compared with the cells without transfection (Figure 6C). In the similar cases, there were no changes for ABCA1 and SREBF1 levels when the cells were transfected with scrambled miRNA when compared with the cells without transfection (Figure 6D). By contrast, miR-33 levels reached the highest level or the lowest level, and were almost same in all groups when the gene was overexpressed (Figure 6E) or silenced (Figure 6G). All the results suggest that LBLP IV from LBL significantly reduces miR-33 level, and relative mRNA level of SREBF1, and increases the level of ABCA1. LBLP IV could not affect the levels of ABCA1 and SREBF1 anymore when miR-33 was overexpressed (Figure 6F, *P* > 0.05) or silenced (Figure 6H, *P* < 0.05). The levels of miR-33 had negative relation with ABCA1 and positive relation with SREBF1 (Figure 6). ABCA1 has negative relation with TG, TC, and LDL-C and positive relation with HDL-C (Figure 6; Table 3). Inversely, SREBF1 had positive relation with TG, TC, and LDL-C and negative relation with HDL-C (Figure 6; Table 3). The results suggest LBLP IV affect the levels of ABCA1 and SREBF1 by regulating miR-33 levels.

The article "Polysaccharide IV from Lycium barbarum L. Improves Lipid Profiles of Gestational Diabetes Mellitus of Pregnancy by Upregulating ABCA1 and Downregulating Sterol Regulatory Element-Binding Transcription 1 via miR-33" was retracted in 2023. Reasons: concerns about the data; concerns about the images.

**Figure 6:** LBLP IV reduces miR-33 level and mRNA level of SREBPF1 and increases the level of ABCA1 in human pancreatic carcinoma cell SW1990. **(A)** The effects of different polysaccharide on miR-33 level. **(B)** The effects of different polysaccharides on relative mRNA levels of ABCA1 and SREBF1. **(C)** The effects of scrambled miRNA on miR-33 level. **(D)** The effects of scrambled miRNA on relative mRNA levels of ABCA1 and SREBF1. **(E)** The effects of miR-33 overexpression on miR-33 level. **(F)** The effects of miR-33 overexpression on relative mRNA levels of ABCA1 and SREBF1. **(G)** The effects of miR-33 silence on miR-33 level. **(H)** The effects of miR-33 silence on relative mRNA levels of ABCA1 and SREBF1. All data were presented as mean values ± SD. There were statistically significant differences if *P < 0.05 and **P < 0.001 vs. a control group.

### LBLP IV from LBL Significantly Reduces Relative Protein Level of SREBPF1, and Increases the Level of ABCA1

Real-time qRT-PCR showed that LBLP I, II, and III reduced while LBL and LBLP IV increased protein levels of ABCA1 (Figure 7A, *P* < 0.05). Comparatively, LBL and LBLP IV reduced relative protein levels of SREBF1 whereas LBLP I, II and III increased the levels of SREBF1 (Figure 7A, *P* < 0.05). All the results suggest that LBLP IV and LBL significantly reduce relative protein level of SREBF1, and increase the level of ABCA1. There were no changes for relative protein level of SREBF1 and ABCA1 when the cells were transfected with scrambled miRNA when compared with the cells without transfection (Figures 7A,B). LBLP IV could not affect the levels of ABCA1 and SREBF1 anymore when miR-33 was overexpressed (Figure 7C, *P* > 0.05) or silenced (Figure 7D, *P* > 0.05). The results suggest LBLP IV affects the protein levels of ABCA1 and SREBF1 by regulating miR-33 level.

The article "Polysaccharide IV from Lycium barbarum L. Improves Lipid Profiles of Gestational Diabetes Mellitus of Pregnancy by Upregulating ABCA1 and Downregulating Sterol Regulatory Element-Binding Transcription 1 via miR-33" was retracted in 2023. Reasons: concerns about the data; concerns about the images.

**Figure 7:** Polysaccharides of *Lycium barbarum L*. (LBLP) IV reduces protein level of sterol regulatory element-binding transcription 1 (SREBPF1) and increases the level of ABCA1 in human pancreatic carcinoma cell SW1990. **(A)** The effects of different polysaccharide on relative protein levels of ABCA1 and SREBF1. **(B)** The effects of scrambled miRNA on protein levels of ABCA1 and SREBF1. **(C)** The effects of miR-33 overexpression on protein levels of ABCA1 and SREBF1. **(D)** The effects of miR-33 silence on protein levels of ABCA1 and SREBF1. All data were presented as mean values ± SD. There were statistically significant differences if *P < 0.05 and **P < 0.001 vs. a control group.

## Discussion

*Lycium barbarum L*. has been reported to have potential anti-inflammatory (45) and anticarcinogenic applications (46), and attenuate lipid peroxidation (47), and diverse health protecting benefits (48). Furthermore, LBLP IV can treat diabetic rats and it can be developed as a potential dietary therapeutic agent in the treatment of diabetes (30). Present findings demonstrate that the LBLP IV is the major compound in LBL and shows significant antidiabetic activities for GDM. More importantly, LBLP IV promotes the insulin secretion (Figure 5), which is beneficial for GDM patients. LBLP IV has been found to reduce serum level of miR-33.

Hepatic mRNA and protein expression of lipid-related genes have been reported to be associated with miRNAs (49). The administration of LBL significantly reduced serum TC and TG levels but increased the HDL-C content (Table 3). The mRNA and protein expression level of ABCA1 were upregulated and SREBF1 was down-regulated (Figures 6 and 7). Furthermore, the expression levels of miR-33, which directly modulate ABCA1 and SREBF1, which indirectly regulates fatty acid synthase (FAS) (50, 51). The repression of miR-33 is a possible molecular mechanism of the hypolipidemic effects of LBLP IV in the liver. Compared with LBLP IV, the three compounds (LBLP I, II, and III) of LBL cannot reduce serum level of miR-33, which regulate ABCA1 and SREBF1, and closely associated with lipid metabolism.

Although LBLP IV was proven to be a bioactive compound from LBL, it could not be made on a large scale. Thus, LBL was still used in subsequent experiment in GDM patients. The changes of biochemical composition indicated that LBL consumption reduced insulin resistance, increased insulin secretory function (Table 2; Figure 5) and improved a lipid profiles (Table 3). Notably, LBL showed a better result after 4 weeks. In contrast, long-term consumption of LBL polysaccharides significantly ameliorates diabetes, including the improvement of general well-being and the decrease of the levels of HbA1c (52), FBG (53), and body mass index (BMI) (54). Similarly, LBL has the functions for controlling the levels of BMI and BG.

The article "Polysaccharide IV from Lycium barbarum L. Improves Lipid Profiles of Gestational Diabetes Mellitus of Pregnancy by Upregulating ABCA1 and Downregulating Sterol Regulatory Element-Binding Transcription 1 via miR-33" was retracted in 2023. Reasons: concerns about the data; concerns about the images.

The reasons for the functions of LBL are complex. According to Chinese theory, LBL can transfer the strength between deficiency and excess from different parts of human body, including upper and lower limbs, internal organs and environment. Full-body and cooperation among different organs are the main ideas of LBL. Differentiation and development genes were repressed by embryonic stem cell-enriched miRNAs, which maintained the stem cell state. MicroRNA level has been reported to be affected by vitamin C (55), polyphenols (56), flavone (57), and polysaccharide (58). Composition analysis of LBL showed that polysaccharides were rich. The results suggest LBLP IV improves antidiabetic capabilities of GDM patients.

Polysaccharides of LBL IV reduced serum level of miR-33, which regulated ABCA1 and SREBP1. The latter two molecules affected lipid metabolism. Thus, LBLP IV improved lipid profiles may by affecting serum miR-33. To approve that, miR-33 was overexpressed and silenced, and the levels of ABCA1 and SREBF1 were significantly changed too (Figures 6 and 7). However, the LBLP IV treatment could not change these molecules anymore. The results suggest that LBLP IV improves lipid profiles by regulating the levels of ABCA1 and SERBF1 *via* miR-33.

The present findings showed that LBLP IV reduced the level of SREBF1 *via* miR-33. The variants of SREBF1 have been found to be discreetly associated with hyperglycemia because of the reduction in insulin sensitivity. SREBF1 is a mediator of insulin action and can affect normal insulin secretion (59). Moreover, the SNP of SREBF1 is closely related to insulin resistance (60). SREBF1 also regulates resistin expression (61). Resistin regulates insulin secretion and glucagon from beta or alpha cells, and pancreatic islets (62). Thus, LBLP IV treatment will affect insulin secretion, HOMA-IR and resistin levels. On the other hand, overexpression of SREBP1 will increase fatty acid synthesis and triacylglycerol accumulation (63) and regulate fatty acid oxidation by activating acetyl coenzyme a carboxylase 2 (64). Although the decrease of SREBF1 can be caused by LBLP-II and –III since the oligosaccharides also regulate miR-33 and the close relationship occurs between miR-33 and SREBF1, the decreased degree was still lower than that caused by LBLP-IV. The result will lead to no significant difference for the changes of lipid profiles when compared with controls.

The article "Polysaccharide IV from Lycium barbarum L. Improves Lipid Profiles of Gestational Diabetes Mellitus of Pregnancy by Upregulating ABCA1 and Downregulating Sterol Regulatory Element-Binding Transcription 1 via miR-33" was retracted in 2023. Reasons: concerns about the data; concerns about the images.

In the past decades, the multitarget of miRNA has caught much interest. miRNA has become a critical factor for regulating lipoprotein (65). Lipid metabolism is a main cause of GDM (66) and there is increasing evidence that miRNA plays an important role in lipid metabolism (67). miRNA can control LDL-C level by regulating TR4 expression in ox-LDL-induced macrophages, and thus affect lipid accumulation (68). miRNA also control LDL-C level by regulating the genes, which are associated with very LDL secretion, cholesterol synthesis, and LDL receptor. Interestingly, several of these miRNAs are located in genomic loci associated with abnormal levels of circulating lipids in humans. MiRNA is a potential drug potential for affecting cholesterol and TG levels in patients (69).

However, the exact molecular mechanism for the effects of LBLP IV on the level of miR-33 remains unknown. There may be the following possible mechanisms: (1) some factors promote microRNA expression by binding miRNA precursor *via* stem-loop recognition (70). LBLP IV may promote microRNA expression by binding miR-33 precursor *via* stem-loop recognition. (2) The relation between amplification and deletion of miRNA binding sites, 3′ UTR length, and miRNA expression has been reported (71). Thus, the site can also be explored to detect the interaction between LBLP IV and miR-33. (3) There is the evidence of the miRNA promoter modification may be a critical determinant of overexpression of miRNA. Restored the hypermethylated promoter can decrease target mRNA and proteins levels (72). Oligosaccharide has an epigenetic effect on gene expression by inhibiting the de-methylation of a “CpG” island within the promoter (73).

There were some limitations to the present study: (1) SW1990 is derived from a spleen metastasis of a grade II pancreatic adenocarcinoma derived from the exocrine pancreas. It is not a representable for a GDM model. A better clinical sample should be applied in this case for analysis. For example, placenta is responsible for transporting nutrients, gasses, and cytokines to the fetu, and eliminate wastes. Thus, normal placental development is very important for the fetus and mother. Trophoblast are the main cells of placenta and primary mouse placental trophoblast cells will be a useful tool to study placental development trophoblast at specific stages of pregnancy (74). Further work shows that Serotonin (5-HT) transporter (SERT) can affect 5-HT concentration in placenta. In GDM, free plasma 5-HT levels are increased because the 5-HT uptake is remarkably reduced, which is caused by impairment in translocating SERT to cell surface. Regular expression of SERT of trophoblast will be beneficial to alleviate GDM-associated complications (75). By using human placenta, the changes of functional SLC6A4 polymorphisms have been found to be associated with long-term outcomes of infants exposed to GDM (76). Insulin signaling is often required for maintaining normal function of SERT on cytoplasma membrane of the trophoblast in placenta. The findings from clinical samples demonstrate that in GDM-associated defect on insulin receptor would change 5-HT uptake rates (77). (2) LBL consumption should be performed in a larger population since the shows little side effects. (3) LBLP IV is the major ingredient in LBL but it is still difficult to determine other components of LBL, which must be determined in the future studies. (4) LBLP IV could not be produced on a larger scale from LBL and LBL was still used in the present study. (5) Some conclusions needed to be confirmed by using broad samples, since only blood serum samples were used in this case. Further work is highly demanded to address these issues.

The article "Polysaccharide IV from Lycium barbarum L. Improves Lipid Profiles of Gestational Diabetes Mellitus of Pregnancy by Upregulating ABCA1 and Downregulating Sterol Regulatory Element-Binding Transcription 1 via miR-33" was retracted in 2023. Reasons: concerns about the data; concerns about the images.

## Conclusion

Long-term LBL consumption was beneficial for improving some symptoms of GDM. However, LBL may have a lot of good or bad effect on GDM because of without the complete examinations for its effects on all aspects or symptoms of GDM. The rehabilitate functions of LBLP IV from LBL may improve lipid profiles. The changes for the level of TG, TC, HDL-C, LDL-C, and MDA also increase antioxidant activity of GDM patients. Furthermore, LBLP IV in LBL plays an important role in antidiabetic activities in GDM patients. Further work is highly demanded to make sure LBL consumption as non-pharmaceutical intervention for preventing the risk or progression of GDM.

## Ethics Statement

All protocols were approved by ethical committee of our hospital (Approval no. 201602X4), and the study was carried out according to the principles described in the World Medical Association Declaration of Helsinki. All subjects gave written informed consent in accordance with the Declaration of Helsinki.

## Author Contributions

SY and LF performed the experiments. LS, WJ, and HP designed the experiment and analyzed all data. RL wrote the article. All authors approved the final submission in this journal.

## Conflict of Interest Statement

The authors declare that the research was conducted in the absence of any commercial or financial relationships that could be construed as a potential conflict of interest.
